# Implementation of Machine Learning Mechanism for Recognising Prostate Cancer through Photoacoustic Signal

**DOI:** 10.1155/2022/6862083

**Published:** 2022-09-20

**Authors:** G. Ramkumar, P. Bhuvaneswari, R. Radhika, S. Saranya, S. Vijayalakshmi, M. Karpagam, Florin Wilfred

**Affiliations:** ^1^Department of Electronics and Communication Engineering, Saveetha School of Engineering SIMATS, Chennai 602 105, Tamil Nadu, India; ^2^Department of Electronics and Communication Engineering, Sri Venkateswara College of Engineering and Technology, Chittoor, Andhra Pradesh 517127, India; ^3^Department of Electronics and Communication Engineering, S.A Engineering College, Chennai 600077, Tamil Nadu, India; ^4^Department of Electronics and Communication Engineering, Easwari Engineering College Ramapuram, Chennai, Tamil Nadu, India; ^5^Department of Electronics and Communication Engineering, Sona College of Technology, Salem 636005, Tamilnadu, India; ^6^Department of Electronics and Communication Engineering, Sri Krishna College of Engineering and Technology, Coimbatore, Tamil Nadu 641008, India; ^7^Department of Electrical, Electronics and Communication Engineering, St. Joseph College of Engineering and Technology, St. Joseph University in Tanzania, Dar es Salaam, Tanzania

## Abstract

Biological tissues may be studied using photoacoustic (PA) spectroscopy, which can yield a wealth of physical and chemical data. However, it is really challenging to directly analyse these tissues because of a lot of data. Data mining techniques can get around this issue. In order to diagnose prostate cancer via PA spectrum assessment, this work describes the machine learning (ML) technique implementation, such as supervised classification and unsupervised hierarchical clustering. The collected PA signals were preprocessed using Pwelch method, and the features are extracted using two methods such as hierarchical cluster and correlation assessment. The extracted features are classified using four ML-methods, namely, Support Vector Machine (SVM), Naïve Bayes (NB), decision tree C4.5, and Linear Discriminant Analysis (LDA). Furthermore, as these components alter throughout the progression of prostate cancer, this study focuses on the composition and distribution of collagen, lipids, and haemoglobin. In diseased tissues compared to normal tissues, there is a stronger correlation between the various chemical components ultrasonic power spectra, suggesting that the microstructural dispersion in tumour tissues has been more uniform. The accuracy of several classifiers used in cancer tissue diagnosis was greater than 94% for all four methods, which is effective than that of benchmark medical methods. Thus, the method shows significant promise for the noninvasive, early detection of severe prostate cancer.

## 1. Introduction

After metastases, prostate cancer has a low chance of being cured and a high occurrence. Prostate cancer was the second highest frequently diagnosed cancer among men globally, as per the 2019 cancer data (following bronchus and lung cancer). Medical imaging detection procedures like ultrasound and magnetic resonance imaging (MRI), which are often used to diagnose prostate cancer, lack data on the chemical makeup of the disease, have low resolution, and are expensive. The high sensitivity, accuracy, and minimum invasiveness requirements for prostate cancer detection are thus still challenging to meet. Checking for increased PSA levels in blood and searching for anomalies during a digital rectal exams (DRE) seem to be the two most prevalent screening procedures for prostate cancer diagnosis. If irregularities were discovered during these testing, the patient can be advised to have a prostate gland biopsy that is guided by transrectal ultrasonography (TRUS). Furthermore, numerous prostate cancer tumours in ultrasound (US) pictures seem to be either isoechoic in origin or resemble other benign prostatic diseases in appearance. A new molecular imaging technique that satisfies the aforementioned characteristics is photoacoustic (PA) spectroscopy. It offers deep acoustic scanning depth over many centimetres and excellent visual contrasts at sub-millimetre pixel size [1]. When a PA signal has been formed, electromagnetic energy acquired by biological tissues has been converted to thermal energy, which causes the tissues' thermal-elastic extension and a localised rise in pressure. After that, the pressure travels as acoustic waves, which are detected by acoustic sensors to create PA signals. Since many biological tissues have distinctive optical absorption spectrum, spectroscopic PA scanning can be used to separate them in a variety of different clinical and research applications. Prostate cancer detection using photoacoustic physio-chemical analysis (PAPCA) has been shown to have tremendous potential. Various bio-macromolecules possess a distinctive light absorption spectrum and can be observed under various light exposures as a result of variations in molecular bonding and vibration modes. The PA signal ultrasonic power spectra can also be used to categorise biological tissues as per their acoustic properties. This approach may concurrently evaluate the prostate tissue's microscopic histologic features and chemical compositions with high resolution and minimal intrusion sensitivity thanks to its optical and ultrasonic properties. In order to advance in this sector, it will be necessary to look into abnormal identification and assessment, create diagnostic tools, and solve the shortcomings of the currently available imaging technology for the prostate cancer diagnosis.

Among the imaging techniques that may be utilised to effectively identify prostate cancer was PA imaging. It was a hybrid imaging method that irradiates soft tissue with pulsed laser light in the near-infrared [NIR] area and measures the US wave the tissue sample emits. The pulsed light was absorbed by the light-absorbing tissue components, resulting in localised heating at the absorbance sites, which would be followed by fast thermal extension and pressure increases. Wide band US waves, commonly referred to as PA waves, are the form in which these pressure increases discharge. US transducers have been used to identify these PA waves, and depending on the applications, various1D signals or 2D grayscale images were created utilising the discovered PA waves. The PA waves' intensity depends on the quantity of light collected by tissue components that, in turn, depends on the tissue's optical absorbance characteristic. The optical absorbance characteristic of the tissue was shown in spatially variable detail in PA pictures created utilising the collected PA waves. The tissue sample's functional information may be obtained via imaging techniques where the picture brightness relies on the optical characteristics of soft tissues. However, one functional data that can be utilised to identify angiogenesis, or the new blood vessel growth, seem to be the spatial variation in tissue's blood content. Malignant lesions are characterised mostly by angiogenesis. By examining the tissue using pulsed laser beams in the NIR frequency area, PA imaging and also conventional optical imaging may be employed to identify angiogenesis. While PA imaging delivers rather acceptable spatial resolution at great depths into soft tissue, simple optical imaging suffers significantly from resolution degradation as the depth within the soft tissue grows. PAPCA was employed for a number of medical detection procedures, including inflammation detection and fibrosis linked to Crohn's illness [2], liver problem assessment [3], bone disorder evaluation [4], microvascular imagery [5], and the prostate cancer detection [6]. Previous research has demonstrated that the PA identification of lipids or haemoglobin could be used to diagnose prostate cancer [7, 8]. Furthermore, the majority of the current study on the possible use of frequency-domain or time-domain PA spectrum in the detection of prostate cancer was concentrated on the physical quantisation factor extraction. This method's accuracy needs to be increased because the information offered by the individual variable extraction for the prostate cancer evaluation has been restricted. The common identification of prostate cancer is shown in Figure 1.

## 2. Machine Learning (ML)

ML seems to be the creation and application of techniques that evaluate the information and its characteristics and, generally, employ statistical methods to select the activities, instead of being expressly designed to allocate particular outputs (behaviour) in accordance to specified inputs (observed environment). Moreover, the creation of methods employing computer programmes that autonomously learns from information and enhances is known as machine learning (ML) [9]. ML techniques were dynamic and frequently get better or “learn” as new data are added. The majority of ML methods can be thought of as statistical frameworks that translate a set of observable variables from a source of data or sampling, known as “predictors” or “features,” into a group of outcome measures, called as “targets” or “labels.” In a procedure referred to as “learning,” the techniques are improved so that they can anticipate the labels by examining the explicit attributes. A sampling would be a digitised slide picture, the features may be the recorded colour intensities of its pixels, and the labelling would have been the Gleason grades ascribed to the tissues in the scanned picture, for instance, in a classification that forecasts the class of prostate tissue's histological imaging. As per the feature type and the label type, ML approaches can be generally categorised. ML can be divided into three categories based on labels: unsupervised, supervised, and reinforcement learning. ML could be divided into nonhandcrafted and handcrafted feature-based methodologies predicted on characteristics. In ML, supervised ML refers to the process of creating a model by teaching computer techniques the link between the input parameters (features) and the outcomes (labels). Before acquiring the input-output connection predicted on the training sample's output labels, the techniques have been first fitted on a training database with the input characteristics. After learning, the techniques have been used to forecast the outcome labels provided the input characteristics on a testing sample's validation database.

### 2.1. Unsupervised Learning

In unsupervised learning, the technique divides the samplings into various classes according to only the characteristics of the training dataset, without assigning matching labels. Samples of such techniques include autoencoders, *k*-means clustering, and principal component analysis for finding collections of related instances in the given data. An approach that recognises distinctive differences of histone changes in immunohistochemically labelled prostate cancer specimens and predicts the likelihood of relapse, regardless of recognised clinical factors like PSA or tumour stage, is an instance of effective unsupervised learning.

### 2.2. Supervised Learning

Expertly labelled relevant databases are the foundation of supervised learning. Engineered feature techniques are taught to reduce forecast error, an assessment of the discrepancy between the known and predicted labels (referred to as the “ground truth”). Naive Bayes classification, support vector machines (SVMs), linear and logistic regression, and random forests are a few instances of such techniques. A great illustration of supervised learning in action seems to be the digitised pathology slide histopathology grading, where pathologists identify the images for noncancer vs prostate cancer and for various Gleason grades. For instance, SVMs could be trained to identify whether newly acquired, unlabelled photos are malignant or benign and to put them on a “cancer likelihood map.”

### 2.3. Reinforcement Learning

A series of methods used in reinforcement learning often run in sequence. On the base of previous and current features, a reinforcement mechanism, or “agent,” reacts on and anticipates the characteristics at each step, and a compensation or penalty was issued based on the forecast. The operator eventually develops a strategy for deciding what to do in each step to maximise the expected yield, which is often the total of anticipated future benefits. A technique that trains to produce the best orientation and amount of operative tissue pullback tension, which supplies counter-forces for robotic scissors or laparoscopy and varies as cutting advances, seems to be an instance of an implementation for like a learning technique. A robotic cutting tool or a laparoscopic operator can use reinforced learning techniques to mechanically provide the right pressure for a particular cutting trajectory.

### 2.4. Nonhandcrafted Characteristics Predicted ML Methods

The raw data are processed as component of the learning procedure in nonhandcrafted characteristic-based approaches. With these techniques, the method “learns” and afterwards adjusts to obtain its own characteristics from the dataset without intentional labelling in order to minimise the forecast error or other classification result measures. These techniques enhance in effectiveness when ever-larger databases have been utilised for training, albeit the resulting characteristics may not always be understandable by humans. Deep learning (DL), which is predicted on artificial neural networks (ANNs) and provides improved problem-solving abilities, is a modern instance of such methods.

### 2.5. Handcrafted Characteristic Predicted ML Approaches

The identification of an infinite number of specific features, which have been prespecified in the database, is a handcrafted feature-based ML approach requirement. The characteristics are predicted on the pertinent data that professionals (such as radiologists or pathologists) normally consider during the diagnosis or decision-making procedure. These distinguishing characteristics are frequently predicted on experienced and professional insights and are susceptible to subjective reasoning. A labelled histology slide's detected glands and nuclei per unit area, as well as their morphology and statistical characteristics, seem to be instances of these specific features. By applying heuristic approaches that adhere to well-known and recognised procedures like edge recognition in image or signal processing, ML strategies requiring a preprocessing phase measure such data in an automatic manner from the sampling.

## 3. ML for Therapy Intervention

Therapy planning and actions can be done using the same ML techniques mentioned for prognostic imaging. Prostate cancer has been found in mpMRI using a feature-enabled ML predictor for external beam radiation therapy (EBRT) and brachytherapy, which had been co-registered with the predicted cancer locations deformable mapping from mpMRI to CT. Then, customised treatment regimens have been created using the expected cancer locations.

## 4. ML in Prognostic Imaging

Interpreting cross-sectional radiographic pictures, like those produced by CT or MRI scanning, basically involves identifying complicated patterns that computers may be learned to do quickly, accurately, and effectively. Low-level computing methodologies, which cope with the pixel classifications for fundamental image assessment tasks like registration, and segmentation, and higher-level methodologies, that provide data like real prostate cancer identification, categorisation, and assessment, are two categories of ML technologies for evaluating virtual prostate images (especially MRI). The low-level classification of approaches has been initially developed using theoretical, analytical, and biomechanical analyses, and then addressed utilising computer vision techniques and image processing, or model-based computations. The spectrum of training data set sizes needed for precise classification varies depending on the ML method and the classes' variability for high-level visual comprehension and assessment. When classifying prostate cancer, handcrafted characteristics need hundreds to thousands of observations, while CNN-based algorithms may need databases 100 times bigger. This criterion does not really automatically imply that it needs thousands of sufferers to learn the techniques, as numerous imaging or pathological regions from any particular patient can be utilised for learning with the necessary “leave-patient-out” evaluation.

The ability to thoroughly evaluate PA physio-chemical spectrum is made possible by the rapid growth of ML. In gene-expression profile assessment, unsupervised ML methods like hierarchical cluster assessment have been frequently employed. These methods demonstrate the huge possibilities of profound data mining by revealing the gene expression's inherent correlations, which are challenging to find explicitly otherwise [10]. By building a categorisation technique for variable optimisation based on training-data examples and labelling, supervised ML techniques, like classification techniques, can significantly increase classification reliability. Clinical uses of ML, such as the detection of breast cancer, brain tumours, and lung cancer, have shown significant promise [11–13]. So, it seems sense that ML may be applied to assess PA spectrum data, as well as enhance the precision of prostate cancer diagnosis.

## 5. Related Works

Some of the recent literatures related to the prostate cancer diagnosis are described as follows.

In ability to forecast prostate cancer using supervised ML, Ismail et al. [14] proposed and verified a number of classification methods. The use of a revised Logistic Regression (LR) classifier on people at risk for prostate cancer has been suggested. The suggested categorisation method makes use of parameters related to the clinical and neoplastic stages. BMI, smoking history, age, and cystitis infections have all been taken into account as clinical factors. In comparison to previous classifiers, the results acquired showed an enhancement in positive prediction value (PPV) and accuracy. Results have been compared and confirmed using sensitivity and specificity effectiveness measures, demonstrating a minimum enhancement in prostate cancer forecast accuracy of 3%. With a 4% enhancement in specificity, the used ML classification algorithm also showed a clinical significance on the prostate cancer identification.

Jović et al. [15] have investigated the feasibility of predicting prostate cancer using ML algorithms. Making appropriate prostate cancer forecasting models is crucial for increasing the likelihood that people with the disease will survive. It is simple to develop an appropriate treatment plan predicted on the pertinent prostate cancer prognosis outcome. Predictive model building is most frequently done using ML approaches. Consequently, a number of machine approaches were used in the investigation and has been compared. The findings were examined and discussed. It was determined that the appropriate prostate cancer forecasting could be done using ML approaches.

Takumi Takeuchi et al. [16] looked at the Deep Learning (DL) effectiveness utilising a multilayer ANN to better precisely anticipate the prostate cancer diagnosis rate on prostatic biopsy. The analysis included 334 participants who received multiparametric magnetic resonance imaging prior to transrectal 12-core prostate biopsy guided by ultrasound. The efficiency of identifying any prostate cancer in testing specimens using learned ANNs with several hidden layers has been around 5–10% greater than that with LR. On input parameters chosen by the sequential LR, the area under the curves (AUC) with multilayered ANN has been considerably bigger than the AUC with LR. The outcome showed that the ANN was only slightly more accurate than LR at predicting prostate cancer without a sample. Nevertheless, ANN performance might still need to be enhanced for clinical application.

Adeel Ahmed Abbasi et al. [17] used transfer learning to create a resilient DL convolutional neural network (CNN). Results have been contrasted using distinct ML tactics (SVM different kernels, Decision Tree, Bayes). A variety of characteristics, including morphological, elliptic Fourier Descriptors, entropy-based, SIFT (Scale Invariant Feature Transform), and texture, are retrieved from the cancer MRI dataset and utilised to train the GoogleNet system and ML algorithms. Different performance metrics like positive predictive value, sensitivity, false positive rate, specificity, receiver operating curve, and negative predictive value are generated for performance assessment. The result indicated that the CNN model (GoogleNet), employing the transfer learning strategy, produced the best results.

The effectiveness of various supervised ML techniques, including k-nearest neighbour, random forest, LR, linear discrimination analysis, linear regression, multi-layer perceptron, SVM, Naive Bayes, deep neural network, and linear classification, for predicting prostate cancer has been contrasted and addressed by Erdem and Bozkurt [18]. This study makes use of 100 patient data from an open-access Internet database on prostate cancer. The outcomes demonstrate that the multi-layer perceptron (MLP) may produce excellent forecasting accuracy that was superior to other methods. According to experimental findings, MLP provides the smallest error rate as 0.03 and the highest accuracy as 97%. The study found that the computer can be medically beneficial with significant accuracy in diagnosing cancer if it is learned using ML techniques predicted on patient data. A patient's invasive biopsy can be avoided in this way.

Irrespective of hand-crafted characteristics, Iqbal et al. [19] have used Residual Net (ResNet-101) and DL long short-term memory (LSTM). Employing non-DL classifiers including SVM, kernel naive Bayes, decision tree (DT), Gaussian Kernel, RUSBoost tree, and k-nearest neighbor-Cosine (KNN - Cosine), the outcomes were contrasted with manually created features like texture, morphology, and grey level co-occurrence matrix (GLCM). This work used ML and DL techniques to minimise the characteristics of cancer images. A jack-knife 10-fold cross-validation procedure has been employed to validate the testing and training data. The outcomes demonstrated that DL ResNet-101 scored better than non-DL techniques and LSTM. Therefore, the ResNet-101 DL approach may be more accurate as a forecast of prostate cancer identification.

Diffusion-weighted magnetic resonance imaging (DWI) was extensively researched for the prostate cancer accurate diagnosis as a component of computer-aided detection (CAD) techniques. Given the deep CNN success in computer vision applications like object segmentation and identification, various CNN architectures are being looked at more and so on in the medical imaging study field as potential solutions for creating more precise CAD techniques for cancer identification. As a result, Yoo et al. [20] devised and put into practise an automatic CNN-based pipeline for axially DWI image- and patient-specific identification of medically relevant prostate cancer. The database, which consisted of 252 and 175 sufferers without and with prostate cancer, was made up of the DWI pictures of 427 people. The result indicated that the presented model has attained higher Confidence Interval (CI).

Due to the existing diagnostic procedure poor performance, such as PSA, digital rectal evaluation, and transrectal traditional US, the prostate cancer (PCa) detection might be difficult. Before biopsy, multiparametric MRI improved PCa identification and has been advised; nonetheless, mp-MRI might miss a significant proportion of PCa. Thus, Correas et al. [21] have developed upgraded micro-US, micro-Doppler, and B-mode procedures and also contrast-improved US and transrectal prostate elastography. These methods can be integrated to create the unique multiparametric US methodology (mp-US). Although mp-US aids in PCa detection, it is not as precise as mp-MRI to completely replace it. In the period of focal treatment, where accurate localisation of PCa has been required, the complementing information provided by mp-MRI and mp-US will become even more crucial.

A NN, which concurrently identifies and classifies cancerous tissues in an end-to-end manner, has been demonstrated by Vente et al. [22]. Contrary to the ProstateX-2 difficulty's categorisation goal, this seems to be more therapeutically relevant. The research trained on and tested against the challenge's database. In this study, brain tumour segmentation patterns that contain the Gleason Grade Group (GGG), a metric for cancer severity, are produced by 2D U-Net, which was fed data from MRI slices. It was also suggested to use the classes' ordinality as a benefit when embedding the GGG in the modelling target and also assess ensembling strategies and ways for using prostate region segmentations as previous knowledge. On the ProstateX-2 challenging testing set, the lesion-wise adjusted kappa has been 0.13 ± 0.27. The outcome showed that the presented strategy goal outperformed multi-label logistic regression and conventional multiclass classification and gave a comparative of techniques for further enhancing the model effectiveness.

A prostate biopsy seems to be a test that determines whether cancer has been present in the tissue or not. Pathologists evaluate whole-slide pictures, which have been created from produced and digitised samples taken from biopsies. These images have a gigapixel quality. Automated intelligence systems may be effective in assisting pathologists with this assessment, easing their workload and accelerating the standard procedure. Therefore, Duran-Lopez et al. [23] introduce a unique DL-based computer-aided detection method. This technology can examine whole-slide histology pictures that have been patch-sampled and preprocessed with various filters, such as a cutting-edge patch-scoring method that eliminates tissue waste. After that, patches are fed into a unique CNN, which outputs a report with a cancerous region heatmap. The computing time required to produce a heatmap for a whole-slide picture was typically 15 seconds. When it comes to operational complexity for a binary categorisation test between healthy and cancerous prostate whole-slide pictures, this unique network performs better than other cutting-edge efforts.

## 6. Materials and Methods

### 6.1. Sample Gathering and Experimental Procedure

The 25 male patients between the ages of 59 and 80, with a mean age of 70.5 years, agreed to take part in the research. Depending on the outcomes of the power research, the patient count was determined. Relying on the outcomes of the PA spectrum's traditional signal processing at 1370 nm and 1210 nm, this study used the software PASS to perform power tests and determine the bare minimal number of samples needed. The slope's average values, predicted on the outcomes at 1370 nm, were −0.059 and 0.073, correspondingly, and the two-sample *T*-test's numerical outcomes under the equal variance assumption are provided in Table 1.

Alternative hypothesis:

(1) $$\begin{array}{c} H_{1}:\gamma =\delta_{1}-\delta_{2}<0\text{.} \end{array}$$

Specifically, two-sample *T*-tests are produced with identical variance. The outcomes are displayed as follows. The average slope readings at 1210 nm are −0.21 and −0.12, correspondingly, and the numerical outcomes for a two-sample *T*-test with equal variation are shown in Table 2. The alternative hypothesis for the 1370 nm and 1210 nm PA spectrum is expressed in (1).

The sample size between 8 and 35 can satisfy the minimum sampling needs, as per the power test findings. As a result, the research gathered as many specimens as it could during the procedure during the past two years, accumulating 25 specimens of prostate tissue. Twenty-two prostate tissue samples from sufferers who had undergone surgery but not prior therapy were used in the investigation, which was carried out in a medical facility. Ex vivo prostates have been surgically extracted, and the blood on their substrates was then cleaned off using sterile gauze. Within one hour of the excision, the tissues have been brought to a PA laboratory at 0°C in an ice bag. Within two hours, the entire PA identification procedure has been finished. Interstitial measures were taken with needle PA probes at 97 different sites under the supervision of skilled medical professionals and predicted on preoperative pathologies. Following the PA measurements, the measurement sites have been marked with a syringe needle. After that, the prostates have been returned to the hospital for a pathological evaluation. Fifty normal areas and 47 malignant sites have been tested, according to the pathology, which is shown in Table 3.

### 6.2. Acquisition of PA Signal

In order to concurrently acquire the PA signals from the specimens and the variant, the experiment's signal collection setup included ultrasonic signal collection and laser triggering. Since the optical wavelength's bandwidth is greater than the typical silicon photodiode's spectrum response range, the research has opted to adjust laser pulse energy using a black body rather than photodiode devices. An adjustable optical adaptive oscillator (OPOTEK, Phocus Mobile, Carlsbad, CA) has been the laser utilised in this investigation. It swept wavelengths between 690–950 nm and 1200–1690 nm at frequencies of 10 nm. Deoxyhaemoglobin, collagen, oxyhaemoglobin, and lipids are among the targeted chromophores that this band was capable of effectively covering. The pulse repetition rate has been 10 Hz, and the pulse width ranged from 2 to 5 ns. The laser beam has been split in the optical axis by a 90 : 10 beam divider, and split light's 10% was then shone on a blackbody. The lenses focussed the 90% split light as well as connected it to a fibre diffuser that we had previously created for laser ablation and had a 300 m radius and a 2 cm length. This study can calculate the laser intensity in mJ/cm^2^ for every wavelength given that the optical energy absorption between the lens subgroup and the fibre coupling had been around 70% and the fibre diffuser's optical outcome area was nearly 0.4 cm^2^.

The input power to the tissue interface has been fulfilled inside the ANSI standard with a maximum of 11.4 mJ/cm^2^ at 720 nm. A needle hydrophone with a bandwidth response of 0–20 MHz (CA, ONDA Corp., HNC1500, Sunnyvale) was used to record the ultrasonic signal produced by the pulsed laser. A centred transducer with a 4.86 MHz central frequency and a −6 dB frequency band of 69.79% (Olympus Corp., Japan, V307-SU, Tokyo) and a pulse receiver with a 1 MHz high-pass filter and 25 dB amplifier (5073PR, Tokyo, Olympus Corp., Japan) have been used to capture the blackbody's ultrasound signals. Here, the significant less frequency noise generated by the dispersed pulsed laser irradiation to the hydrophone's surface has been suppressed using a 1 MHz high-pass filtering. After that, the information was gathered with an oscilloscope (Tektronix, TDS 3034B, USA, Ohio) and saved in a pc (ThinkPad S3 5440, Lenovo, China). To get a good signal-to-noise ratios, the signal was averaged 128 times (SNR) and also created a programme to autonomously change the wavelength roughly every 15 s using the 10 pulses/second laser's frequency.

### 6.3. PA Physio-Chemical Spectrum

In this paper, the data processing approach was first used. The tissue's time-domain signal has been dividing the blackbody signal's peak-to-peak value tissues, and the tissue signal's laser energy has been corrected. The PA signal's power spectrum was then measured using MATLAB R2020a and the Welch technique. For the window's sliding computation, the research by default employed Hamming windows with a 2500 sample point's length and 90% overlap. The hydrophone has 0–20 MHz frequency response range. The analysis frequency range has been found to be 1–20 MHz following applying a 1 MHz high-pass filtering and a 0.1 MHz frequency spectral resolution. The observed power spectra that corresponded to the wavelengths were arranged to produce the PA physio-chemical spectra. The PA signal's intensity spectrum, which indicated the PA source's content, has been generated by aggregating the power spectrum at PA physio-chemical spectrum's various wavelengths. The spectra's characteristics are then examined using ML techniques. The layout of the presented framework is shown in Figure 2.

### 6.4. Hierarchical Clustering and Pearson Correlation-Coefficients (PCCs) Map

A total of 77 wavelengths have been designated from 0 to 76 according to size (1200–1690 nm, 690–950 nm, Δ*λ* = 10 nm). Baidu's open-source visualisation platform, Echarts, was used to build all ML calculations and visualisations. The Pearson correlation coefficients (PCCs) for the various wavelength power spectra were determined via the Python Pandas. The wavelength's power spectrum was thus combined to form the PCC matrix. The matrix had 77 × 77 dimensioned (a symmetric diagonal matrix). The PCC matrix has been subjected to a cluster analysis using an unweighted pair grouping technique with arithmetic mean (UPGMA), and the correlation-coefficient matrix has been acquired after clustering. Six groups made up the clustered group. The PCC matrix for every sample point was present.

With the usages of further statistical evaluation and visualisation, this research employed the correlation-coefficient network architecture to more clearly see and understand the distinctions between healthy and malignant prostate tissues. In this case, 77 wavelengths (1200–1690 nm, 690–950 nm, Δ*λ* = 10 nm) have been viewed as 77 nodes, and they have been all dispersed around a circle. Additionally, the percentage of specimens in this group's overall sample size with correlation coefficients *R* larger than 0.9 for each pair of wavelengths was determined. The correlation weight WR has been used to describe the proportion variable. Also placed a line among the nodes designating between two wavelengths when those wavelengths WR were greater than 70%. The related correlation-coefficient network architecture was created after calculating the WRs for each wavelength. Three indicators have been utilised in the correlation-coefficient network architecture to depict the variations in correlation:

- Node size: if there are more connections in node, its size is larger
- Connectivity: when WR is greater than 0.7, the connectivity among the nodes exists
- Label of node (optional): if node size > threshold, the node label has been added

All samples were separated into healthy and tumour groups, the two group's correlation-coefficient network was computed, and the findings were shown.

## 7. Prostate Cancer Classification

In this research, three methods were used to classify the prostate cancer, i.e., SVM, Naïve Bayes (NB), C4.5, and Linear Discriminant Analysis (LDA).

### 7.1. Naïve Bayes (NB)

In prostate cancer classification, an ML approach known as Naïve Bayes (NB) is used. The NB theorem has been used to create probabilistic classifiers called NB. In terms of prostate cancer classification, NB is a simple and effective method. The fact that NB is a highly scalable algorithm is one of its key features. Simply put, the NB classifier posits that the presence of some characteristics in a class has no bearing on the presence of any other characteristics. This theory has been adopted in evaluating the prostate cancer on

(2) $$\begin{array}{c} Q^{*}={argmax}_{Q}P\left(\frac{Q}{D}\right)\text{,} \end{array}$$

(3) $$\begin{array}{c} Q^{*}={argmax}_{Q}P\left(\frac{Q}{D}\right)\times \left(\frac{P\left(Q\right)}{P\left(D\right)}\right)\text{,} \end{array}$$

where *Q* is the prostate tissue and *D* is the normal. This classification method looks at the relationship among each characteristic and each feature in a signal, presuming that all characteristic values were absolutely independent. It evaluates each feature individually and calculates a conditional probability for the relationships between the cancer tissues and normal. As the anticipated cancer, the category with the greatest probability score is chosen.

### 7.2. Support Vector Machine (SVM)

Among the popular classifiers, the commonly used one is support vector machines (SVMs). SVMs are among the strategies used in supervised ML. SVMs employ a training technique to create a classifier, which will be employed to allocate new unknown parts to one of many predetermined categories. SVMs could be utilised to classify data in both linear and nonlinear ways. SVMs could also be used for both supervised and unsupervised learning. SVMs produce a hyperplane or a series of hyperplanes, which are then employed for classification. Moreover, in SVMs, the classes are in the form of hyperlane, which is shown in

(4) $$\begin{array}{c} S.G+b=0\text{,} \end{array}$$

where *S* is the vector's weight, *G* is the input vector, and *b* denotes bias.

### 7.3. Decision Tree (C4.5)

A decision tree appears to be a prediction framework in learning. A decision tree's main objective was to incorporate a framework that could anticipate the value of the target parameter. In such a decision tree, the variables created during the training phase have been used to forecast the targeted variables. One of the simplest classification models was a decision tree. A decision tree uses clear and basic concepts to solve classification problems. A decision tree often consisted of a number of attributes. Decision trees come in several forms, including ID3 and C4.5.

The ID3 decision tree-based strategy, which constructs the tree top-down, appears to be improved by C4.5. The conquer-and-divide method, which divides the input vector into local areas based on a distance metric, is used to construct a decision tree. The roots and intermediary nodes' attributes are chosen using information theory. Starting at the root node and iterating through the process until leaf nodes are located, the C4.5 approach builds a decision tree. One of the best data mining classifiers is C4.5. C4.5 appears to be a statistical system of classification. The decision tree is built by C4.5 from a collection of training databases. Based on knowledge growth and gain ratio, C4.5 ranks potential exams. C4.5 is made up of four stages, which are detailed as follows:

1. Assign a feature as a root
2. Create a branch for each value
3. Put database in branch
4. Continue the second step until all of the classes have the similar value

Formulas employed in C4.5 method is represented in

(5) $$\begin{array}{c} V=\sum_{i=1}^{n}-P_{i}\times \log_{2}P_{i}\text{,} \end{array}$$

where *V* denotes entropy, and *P* denotes the proportion of class in the output.

(6) $$\begin{array}{c} Gain\left(V,F\right)=S\times \sum_{i=1}^{n}\left(\frac{\left|V_{i}\right|}{\left|V\right|}\right)\times V\text{,} \end{array}$$

where *V* is the set of case, *F* is the case attribute, |*V*_*i*_| is the number of cases to iteration *i*, and |*V*| represents the number of cases in the set.

### 7.4. Linear Discriminant Analysis (LDA)

A two-dimensional matrix with 77 wavelengths (1200–1690 nm, 690–950 nm, Δ*λ* = 10 nm) and frequency points of 191(1–20 MHz, Δ*f* = 0.1 MHz) made up the raw PA physio-chemical spectra. By computing one-dimensional matrices among classes and condensing these one-dimensional matrices to a unique numerical value, referred to as the mapping valuation, LDA has been utilised to resolve the dichotomy issue. In this work, the initial 77-component one-dimensional matrices have been taken into consideration, and using LDA, it has been minimised to a unique value using the single frequency point's power-values at various wavelengths. Healthy and malignant tissues might be distinguished by the appropriate mapping number being higher than zero after this mapping number was normalised. Additionally, predicted on the computed preset values, all frequency points' mapping values were computed in anticipation, and the frequency points that could definitively distinguish between healthy and tumour samples were extracted. The ultimate prostate cancer prognosis was made using these frequency-point mapping mean values as eigenvalues. Ninety samples have been randomly chosen from a pool of 97 data for the classification test in order to train an acceptable linear mapping. The model was tested using the remaining seven examples.

The test set seems to be quite tiny for a solitary holding out set, wherein 90% of the information has been employed for training and 10% have been employed for testing. As a consequence, there are significant differences in the effectiveness estimates for various data samples or for various ways to divide the data into testing and training sets. In this experiment, the 10-fold cross-validation calculation has been carried out and split the information into 10 categories, only one of which was employed for testing. Every divided group was then evaluated as a test set. Also, using the k-fold cross-validation, *k* LDA method was trained, and thus able to calculate all model's average accuracy. The variance has been decreased by averaging over *k* distinct partitions, which lessens the performance estimate's sensitivity to the data splitting. As a result, the model's resilience is assured. There is no set formula for choosing *k*. According to Ron Kohavi's cross-validation research, a 10-fold cross-validation has been selected for its objectivity and less variance. To determine the final model's correctness, the model underwent 10-fold cross-validation that was performed three times. The mean value has then been determined.

### 7.5. Statistical Analysis

The intercept and slope have been recovered as the traditional quantification variables for prostate cancer detection using the usual PA spectrum assessment techniques. For a relevance analysis, a one-sided *P*-value of under 0.05 has been used. The area under cure (AUC) was then computed to evaluate the effectiveness of ML with traditional analysis techniques. All AUC calculations were made using Python (3.7) and GraphPad Prism, while Matlab has been used to extract the standard quantification variables.

## 8. Evaluation Metrics

The effectiveness of prostate cancer detection is evaluated using well-established criteria, enabling for contrast with existing approaches. A number of factors, including the system's operation, influence the selection of an appropriate evaluation metric. Furthermore, evaluation measures are critical in assessing the outputs of classification models. In this study, the presented model evaluated the outcomes using sensitivity, accuracy, and specificity.

### 8.1. Accuracy

The ratio among the number of cancer that were accurately classified and the total number of texts is known as accuracy. To assess the effectiveness of the learning techniques, accuracy has been employed as an evaluation metrics for prostate cancer detection. The accuracy metric measures the overall number of flows identified properly across all classes.

Accuracy is computed by

(7) $$\begin{array}{c} accuracy=\frac{T_{P}}{T_{N}}\text{,} \end{array}$$

where *T*_*N*_ denotes the number of input samples that are not assigned to a certain class. *T*_*P*_ represents the number of corrected predictions in a given class that are appropriately identified.

### 8.2. Specificity

Specificity is described as the number of cancer tissues accurately allocated to class divided by the overall number of cancer patients genuinely belonging to class.

Specificity is computed by

(8) $$\begin{array}{c} specificity=\frac{no.\;of\;correctly\;classified\;cancers}{total\;number\;of\;input\;cancer\;samples}\text{.} \end{array}$$

### 8.3. Sensitivity

The ratio of the number of cancerous tissues accurately categorised as pertaining to class to the overall number of input samples as pertaining to class is referred to as sensitivity. Sensitivity is indeed an important parameter of cancer classification outcomes because it is delicate to inaccurate classification. Moreover, inaccurate categorisation resulted in less sensitivity results.

Sensitivity is computed by

(9) $$\begin{array}{c} sensitivity=\frac{no.\;of\;accurately\;predi\;cted\;cancer}{overall\;number\;of\;input\;cancer\;samples}\text{.} \end{array}$$

## 9. Results and Discussion

### 9.1. Prostate Tissue's PA Physio-Chemical Spectrum

To produce the actual PA physio-chemical spectra, the obtained PA power spectrum has been organised by wavelength. The spectra show the variations between healthy and malignant tissues. The cancerous tissues PA physio-chemical signal in both areas is much greater than that of healthy tissues (orange dashed box). Haemoglobin seems to be the principal light and sound generator in the 680–940 nm region. Due to the blood vessels' obvious growth during the progression of cancer, tumour tissues have a higher overall haemoglobin content, which causes their colour to be noticeably greater than that of healthy tissue. Lipids and collagen seem to be the principal sources of PA in the range of 1200–1370 nm. Their signals are often greatly improved, showing that the prostate tissue's collagen and lipid concentration rises during carcinogenesis. By contrasting the PA signal intensity spectrum with the light-absorption spectrum of other biomolecules, signal amplification in such two locations may be seen more vividly.

### 9.2. Prostate Tissue Biomacromolecule Correlation Assessment via PA Physio-Chemical Spectra

For academics in the domains of cluster and taxonomy analysis, utilising points of varied colouring to reflect closeness and actual data matrix is not unique, and it has proven effective for acquiring better architecture or restoring lost structure. Utilizing UPGMA and PCCs, the 77 wavelengths have been divided into six wavelength categories. The biomolecule light-absorption spectra have been then contrasted to the clustering outcomes. The cluster tree's 77 terminal nodes have not been ordered in the sequence 0–76, but the wavelength clustering is quite similar to the collection of distinct biological macromolecules that absorb light. Furthermore, due to variations in molecular bonding and vibration patterns, various biomacromolecules exhibit distinct light-absorption spectrum. The detecting wavelength bands, wherein the PA signals produced by various biomacromolecules predominate, are defined by UPGMA, which also aids in analysing the variations in PA spectra. These are the groups: deoxyhaemoglobin (W1) (#0–12; 680–790 nm); oxyhaemoglobin (W2) (#13–25; 800–940 nm); lipid 1 (W3) (#26–33; 1200–1250 nm); collagen (W4) (#34–48; 1260–1390 nm); water (W5) (#49–72; 1400–1640 nm); and lipid 6 (W6) (#73–78; 1650–1680 nm). All tissues test wavelength clustering outcomes have been statistically examined.

Because the primary biomolecules in healthy or cancerous cells were the same, no discernible variation in clustering outcomes between healthy specimens and cancerous ones has been found. The numerous pseudo-colour intensities represented the different chemical group's intergroup and intragroup correlation coefficients. Also, this model combined (W3–W6) for presenting the analyses because although the group's relative locations differed during the UPGMA clustering procedure, the results have been unaffected. Since the vascular system remained distinct from the other element's distribution, the vascular correlation groupings (W1–W2) from these specimens displayed a minimal correlation with some other groupings (W3–W6). The intergroup association between W1–W2 as well as W3–W6 has also been found to be higher (the colour was deeper) in the malignant tissues when we compared the healthy and cancer specimens. W1 and W2 have been grouped together as a result of their strong association. The network maps displaying all test statistical outcomes make this correlation extremely clearer. This research may observe an enhancement in the connection between various groups for all three of the aforementioned indicators:

1. Malignant tissues have more edges than healthy tissues in their network maps
2. The cancerous-tissue networking map shows significantly larger nodes
3. The malignant tissue network map has more labels

The microstructural alterations of these two biological macromolecules with the progression of prostate cancer make the association between collagens and lipids more obvious than before. Adequate structural support for prostate tissues has been provided by collagen fibres, and the cell membrane primary elements in external exosomes were lipids. They have various distribution systems since they are dispersed around the organisation in various locations. Nevertheless, the environment transforms and metabolism seems to be irregular when prostate tissues become malignant. The diverse tumour environment makes the PA spectra more diverse and muddles the particular substance's distribution properties, enhancing the PA spectrum's connection.

Wavelengths might be categorised predicted on power similarities using cluster and correlation analysis, providing a precise reference for identifying various cellular macromolecules. The aforementioned analysis also demonstrates that the differences in the bio-macromolecule's microstructure that occur during the prostate cancer evolution can be accurately reflected by the PA physio-chemical spectra, demonstrating the effectiveness and viability of diagnosing prostate cancer using the PA physio-chemical spectra.

### 9.3. Prostate Cancer Identification through SVM, NB, C4.5, and LDA

The correlation-coefficient map's overall correlation is significantly greater (>0.75), implying that redundant data have been present, despite the cluster and correlation assessments showing that the PA physio-chemical spectra can accurately reflect the various biological macromolecule microstructural changes. The categorisation problem cannot be solved given the high correlations. Prostate cancer detection is primarily a binary categorisation challenge of separating malignant tissues from healthy tissues. In order to eliminate unnecessary data in the wavelength dimensions, extract variables that may more accurately reflect tumour features, and increase diagnostic precision, this research used LDA, SVM, NB, and C4.5 methods. In order to investigate the 97 data distribution, this study determined the mapping values for all 97 data under these ML-models after training the LDA modelled at various frequency points. Two basic distributions existed in the data's mapping-value distribution depending on the LDA that was acquired by training at various intensity points. The last 47 specimens have been tumour samples, while the first 50 specimens had been healthy samples. In the first distributions, a threshold allowed a complete separation between the estimated mapping values of the healthy sample and the tumour sample's predefined value. There has been no threshold that could totally separate the tumour samples from the healthy sample. It is evident that the frequency points of mapping-value distributions without overlapped regions performed better at differentiating between healthy and malignant samples. The differences in data attributes are the apparent cause of the efficiency differences between distinct frequencies. Finding a linear mapping may maximise the variation between categories and minimise the variation within categories, as per the theory behind the LDA method, resulting in target differentiation. Due to the varied data characteristics at these two frequency intervals, LDA can discriminate between them to varying degrees.

The main cause is that our targeted chromophore size varies depending on the frequency range and that chromophore dimensions affect how well the model can characterise or describe diseased traits. As a result, in order to increase the diagnostic precision, combination assessment approach has been used, which called for using the average value of the estimated mapping variables at these frequency intervals as the ultimate categorisation eigenvalue.  Table 4 lists the chosen frequency points and prostate cancer diagnosis made using just those frequencies. The combined evaluation also showed that, after 10-fold cross-validation, done three times for 97 samples, the average reliability could reach 95.8 percent. This accuracy rate has been comparable to that of methods frequently employed in clinical settings; multi-mode ultrasound (US) has an accuracy of roughly 71.7% [24], while MRI has attained an 80% accuracy for diagnostic purposes [25]. As a result, PA spectroscopy's efficiency for diagnosing prostate cancer using the LDA technique is on par with that of US and MRI. According to theory, LDA is more effective at categorising data when the correlation matrix would be the same. Hence, it is logical to assume that as data accumulates, its properties, particularly the covariance matrices, would become clearer and the analytical upper range that LDA may accomplish will be more easily determined.

With more information, a more efficient linear mapping with the lowest intra-class variation and highest inter-class variance could be established, further increasing the prognostic accuracy. As a result, the LDA would reach its upper limit of judgement if there are appreciable changes in the characteristic distribution's covariance matrix between healthy samples and tumour samples in the gathered information. LDA was appropriate for categorisation of small samples.

Multidimensional variables can be limited to a single number for categorisation if the variables are assumed to be linear and the progression of the illness is linear. In actuality, there may be nonlinear relationships between the physio-chemical spectra of PA and tumour development. Moreover, the diagnostic accuracy of other three models has also attained higher rates. The overall outcome of the presented model is shown in Table 5 and Figure 3. Further, the outcome of the presented method's accuracy was compared with other prostate cancer diagnosis methods, as shown in Table 6 and Figure 4.

## 10. Conclusion

In this study, diagnostic algorithms for prostate cancer were developed using the PA physio-chemical spectrum of healthy and malignant prostate tissues. Also, the correlations between various macromolecules in healthy and malignant tissues using the UPGMA cluster analytical technique were compared, and thus the distinctive light-absorption regions, W1–W6, of various biological macromolecules were identified. As per the healthy and tumour sample visualisation results of W1–W6, it was discovered that the haemoglobin, collagen, and lipid power-spectrum correlations have been significantly higher for malignant prostate tissues than for ordinary prostate tissues, representing a rise in the microstructural resemblance of the dispersion of these biological molecules. Moreover, this research uses four methods for diagnosing prostate cancer, namely, SVM, C4.5, NB, and LDA. The presented models have attained higher accuracy rates, i.e., LDA has attained a 95.8% accuracy, NB acquired a 95.2% accuracy, C4.5 earned a 97.3% accuracy, and SVM has attained a 96.8% accuracy. The findings of this work demonstrate the viability and efficiency of using ML and PA physio-chemical spectroscopy in conjunction to explore the differences in the microscopic architecture and chemical makeup of prostate cancer and hence facilitate its identification. To further increase the diagnosis accuracy, more data should be gathered and the classification method should be further refined. The categorisation should also discriminate between benign and malignant tumours to improve the method's practical applicability.

## Figures and Tables

**Figure 1:** Prostate cancer identification process.

**Figure 2:** Presented framework.

**Figure 3:** ML-methods overall outcome.

**Figure 4:** Accuracy comparison.

**Table 1:** Outcome of power study predicted on 1370 nm PA power spectrum slopes.

AP	TP	*δ*_1_	*δ*_2_	*γ*	*N *_1_	*N *_2_	Alpha	*σ*
0.71	0.7	−0.3	−0.2	−0.1	12	12	0.01	0.1
0.80	0.8	−0.3	−0.2	−0.1	14	14	0.01	0.1
0.92	0.9	−0.3	−0.2	−0.1	18	18	0.01	0.1
0.76	0.7	−0.3	−0.2	−0.1	8	8	0.05	0.1
0.81	0.8	−0.3	−0.2	−0.1	9	9	0.05	0.1
0.91	0.9	−0.3	−0.2	−0.1	12	12	0.05	0.1

*Note.* AP, actual power; TP, targeted power.

**Table 2:** Outcome of power study predicted on 1210 nm PA power spectrum slopes.

AP	TP	*δ*_1_	*δ*_2_	*γ*	N_1_	N_2_	Alpha	*σ*
0.72	0.7	−0.3	−0.2	−0.1	25	25	0.01	0.1
0.81	0.8	−0.3	−0.2	−0.1	28	28	0.01	0.1
0.90	0.9	−0.3	−0.2	−0.1	35	35	0.01	0.1
0.71	0.7	−0.3	−0.2	−0.1	14	14	0.05	0.1
0.80	0.8	−0.3	−0.2	−0.1	17	17	0.05	0.1
0.90	0.9	−0.3	−0.2	−0.1	25	25	0.05	0.1

*Note.* AP, actual power; TP, targeted power.

**Table 3:** Radical prostatectomy's 97 samples from whole prostate-25 cases.

Prostate	PA-measurement	PP	*P*N	WPP
1	3	2	1	B
2	2	1	1	B
3	4	2	2	B
4	3	1	2	B
5	5	3	2	B
6	5	4	1	B
7	3	2	1	B
8	5	0	5	C
9	4	3	1	B
10	5	3	2	B
11	4	2	2	B
12	6	0	6	C
13	3	1	2	B
14	4	3	1	B
15	6	4	2	B
16	3	0	3	C
17	6	4	2	B
18	3	1	2	B
19	2	1	1	B
20	3	2	1	B
21	5	0	5	C
22	4	3	1	B
23	3	2	1	B
24	2	1	1	B
25	4	2	2	B
Total	97	47	50	

*Note.* PP: pathologically positive, PN: pathologically negative, WPP: whole prostate pathology, B: aggressive, and C: nonaggressive tissue.

**Table 4:** Accumulative prediction outcomes based on frequency selection.

FSM	*F* (MHz)	SFFA (%)	AFFA (%)
All specimens have been completely differentiated from healthy and cancer samples	2.8	92.4	95.8
	6.1	94.6	
	8.1	91.3	
	9.9	96.5	
	12.9	95.4	
	15.4	92.8	
	16.1	95.25	
	18.3	95.7	

*Note.* FSM: frequency selection method, F: frequency, SFFA: single frequency forecasting accuracy, and AFFA: assembled frequency forecasting accuracy.

**Table 5:** Overall outcome.

Method	Sensitivity (%)	Specificity (%)	Accuracy (%)
SVM	93.4	94.4	96.8
NB	95.1	92.9	95.2
C4.5	92.8	91.5	97.3

**Table 6:** Comparison of accuracy.

Methods	Accuracy (%)
US	71.7
MRI	80
LDA (PA)	95.8
C4.5 (PA)	97.3
NB (PA)	95.2
SVM (PA)	96.8

## Data Availability

The data used to support the findings of this study are included within the article.
